The article "Determinants of Hypertension Among Patients With Type 2 Diabetes Mellitus in Karachi, Pakistan: A Cross-Sectional Study" was retracted in 2022. Reasons: false authorship; lack of ethics approval or compliance; concerns about the data; concerns about the authorship.

# Determinants of Hypertension Among Patients With Type 2 Diabetes Mellitus in Karachi, Pakistan: A Cross-Sectional Study

**DOI:** 10.7759/cureus.22157

**Published:** 2022-02-12

**Authors:** Chamithra D Rupasinghe, Usama Shahbaz, Ellen Huang, Akshay Patel, Fares Mohammed Saeed Muthanna, Marina Basta, Chutimon Narawish, Sehrish Karim, Anum Rahim

**Affiliations:** 1 Internal Medicine, Manipal College of Medical Sciences, Pokhara, NPL; 2 Clinical Sciences, Saint James School of Medicine, The Quarter, AIA; 3 Internal Medicine, Oceania University of Medicine, Apia, WSM; 4 Internal Medicine, Saint James School of Medicine, The Quarter, AIA; 5 Pharmaceutical Care, Walailak University, Nakhon Si Thammarat, THA; 6 School of Medicine, St. George's University, True Blue, GRD; 7 College of Medicine, Rangsit University, Pathum Thani, THA; 8 Public Health Sciences, Aga Khan University Hospital, Karachi, PAK; 9 Indus Hospital Research Center, The Indus Hospital, Karachi, PAK

**Keywords:** pakistan, prevalence, determinants, type 2 diabetes mellitus, hypertension

## Abstract

Introduction: Hypertension is the persistent rise of systemic arterial blood pressure. Among diabetic patients, hypertension is one of the important public health challenges. The frequency of hypertension among diabetic patients is almost twice than that of non-diabetic patients. This study aims to determine the determinants of hypertension among type 2 diabetes patients in Karachi, Pakistan.

Methodology: This was a cross-sectional study conducted in diabetic clinics of a tertiary care hospital from August 2020 to August 2021. The source population included all adult patients with type 2 diabetes at the follow-up clinic of Liaquat National Hospital and Aga Khan Hospital. Data collection was done using a structured interviewer-administered questionnaire. REDCap software (Vanderbilt University, Nashville, TN) was used for the data collection.

Results: A total of 610 patients were included in the study. The mean age of participants was 57.37 (±11.32) years. The overall prevalence of hypertension among diabetic patients was 39.84%. Age, physical activity, family history of hypertension, smoking status, BMI, sedentary lifestyle, stress level, and serum creatinine were independent determinants of hypertension among people with type 2 diabetes mellitus.

Conclusion: In this study, age, physical activity, family history of hypertension, smoking status, BMI, sedentary lifestyle, stress level, and serum creatinine are independent determinants of hypertension among type 2 diabetes patients. The findings of the study call for strategies that can target these predictors, and clinicians need to start educating their patients about hypertension and ways to prevent it.

The article "Determinants of Hypertension Among Patients With Type 2 Diabetes Mellitus in Karachi, Pakistan: A Cross-Sectional Study" was retracted in 2022. Reasons: false authorship; lack of ethics approval or compliance; concerns about the data; concerns about the authorship.

## Introduction

The persistent rise in systemic arterial blood pressure (BP) is known as hypertension. There is no sharp differentiation between normal BP and hypertension. Still, for clinical reasons, it is defined as systolic blood pressure (SBP) of 140 mmHg and/or diastolic blood pressure (DBP) of 90 mmHg, or any prior diagnosis of hypertension made by a healthcare professional, and the use of antihypertensive medications [1]. Among diabetic patients, hypertension is one of the important public health challenges [2]. The frequency of hypertension among diabetic patients is almost twice as compared to non-diabetic patients [3]. The presence of hypertension in diabetic patients increases the risk of cardiovascular events and death by 41% and 44%, respectively, compared to 9% and 7% in those with diabetes alone [4]. Hypertension is thought to be responsible for 7.5 million deaths per year, 57 million disability-adjusted life years, and around 6% of all deaths in the world [5]. Nearly one billion individuals worldwide suffer from hypertension, with two-thirds living in developing nations [6].

Preventing hypertension is more beneficial than treating it, especially among diabetes patients, as it will cause systemic malfunctioning that is tough to manage [7]. Preventing hypertension also aligns with one of the three goals of the Global Action Plan of the World Health Organization (WHO), which targets a 25% relative reduction in hypertension prevalence [8]. However, more evidence on the predictors of hypertension is needed for successful disease prevention and its harmful repercussions, particularly among the diabetic population. The risk factors for hypertension may differ from those in the general population.

For individuals with type 2 diabetes, complete cardiovascular risk assessment, management, and counseling are an important part of disease management [9] as a large number of diabetic patients (>68%) die due to cardiac complications [10]. In addition to the increased risk of death from cardiovascular disease (CVD) in diabetic patients, hypertension increases the risk of CVD-related death in type 2 diabetes patients [9]. Because hypertension is one of the most common risk factors for CVD in this population, understanding its causes is critical for preventing and controlling CVD and other complications of diabetes mellitus [11].

Identification of the determinants of hypertension among type 2 diabetes patients will enable healthcare professionals to tackle its impacts on patients effectively. Besides this, it can also help policymakers design appropriate strategies for reducing health-related costs. There is currently no documented evidence in Pakistan about the factors of hypertension in diabetes patients. Therefore, the current study has been conducted to determine the determinants of hypertension among type 2 diabetes patients in Karachi, Pakistan. The current study will provide data related to the magnitude of hypertension along with its determinants among type 2 diabetes patients for planning for investigations.

The article "Determinants of Hypertension Among Patients With Type 2 Diabetes Mellitus in Karachi, Pakistan: A Cross-Sectional Study" was retracted in 2022. Reasons: false authorship; lack of ethics approval or compliance; concerns about the data; concerns about the authorship.

## Materials and methods

Methodology

This was a cross-sectional study conducted in diabetic clinics in a tertiary care hospital from August 2020 to August 2021. The source population included all adult patients with type 2 diabetes at the follow-up clinic of Liaquat National Hospital and Aga Khan Hospital. The study population included all patients with type 2 diabetes who were under routine follow-up at the above-mentioned hospitals during the period of data collection. The ethical approval of this study was taken from Liaquat National Hospital ethical review committee (IRB number: LNH_2020_07_05).

Eligibility criteria

The study included type 2 diabetes patients who had at least one prior visit and were at least 18 years old. The study excluded pregnant women and patients whose hypertension diagnosis came before their type 2 diabetes mellitus diagnosis. Besides this, critically ill patients having a cognitive impairment that affects their ability to give responses and hearing difficulty were also excluded from the study. Type 2 diabetes patients with hypertension were taken as cases, while type 2 diabetes patients without hypertension were considered as controls.

Sample size and sampling technique

The sample size was calculated using a single population proportion formula by taking the overall prevalence of hypertension among diabetic patients, i.e., 37.4% [12], 95% confidence interval, and 5% margin of error. This gives a sample size of 605. Participants were enrolled using a non-probability consecutive sampling technique. Patients with type 2 diabetes who visited the hospital for a follow-up during the study duration were invited to be a part of the study. Patients were enrolled in the study until the desired sample size was achieved.

Data collection procedure

Data collection was done using a structured interviewer-administered questionnaire. REDCap software (Vanderbilt University, Nashville, TN) was used for the data collection. Behavioral variables were assessed using the WHO stepwise approach for risk factor surveillance of chronic disease [12]. Three third-year nursing students were recruited for the data collection, and training was given to them related to the data collection instrument and software. Before proceeding with data collection, a pretest of the questionnaire was done on 25 type 2 diabetes patients who were not part of actual data collection and final analysis.

The article "Determinants of Hypertension Among Patients With Type 2 Diabetes Mellitus in Karachi, Pakistan: A Cross-Sectional Study" was retracted in 2022. Reasons: false authorship; lack of ethics approval or compliance; concerns about the data; concerns about the authorship.

To measure the level of stress of patients, Cohen’s 10-item Perceived Stress Scale (PSS) was used [13]. Data related to laboratory and clinical profiles of participants were obtained from the hospital management information system (HMIS). Data obtained from HMIS included hemoglobin A1c (HA1C), serum creatinine, high-density lipoprotein (HDL), low-density lipoprotein (LDL), and total cholesterol.

Measurements

Following standard procedure, BP was taken with a mercury sphygmomanometer (adult size). After the patient had rested for at least five minutes, BP was taken from the left arm in a sitting position with feet on the floor and arm supported at heart level. Patients who had consumed coffee in the hour before the measurement or who had smoked in the 30 minutes before the measurement were allowed to stay for at least one hour and 30 minutes, respectively, from the time of those events.

International Physical Activity Questionnaire - Short Form (IPAQ-SF) was used to assess the physical activity level. It estimates the total level of physical activity of an individual in metabolic equivalent (MET)-minutes/week by the number of days in one week and determines the duration in minutes in engagement in three types of activity, including high-intensity activities, moderate-intensity activities, and walking in the last seven days. Participants were classified into three levels of physical activity, including low, moderate, or high as per the cutoff of total MET-minutes/week in each category [14].

Individuals were classified sedentary if they reported reclining or sitting for more than four hours at work, home, on public transportation, or with friends, but not including time spent on sleeping. A portable weight machine was used to measure body weight to an accuracy of 0.1 kg. Participants wore light indoor clothing and were barefoot. Standing upright on a flat surface, height was measured with a stadiometer in meters. The ratio of weight in kilograms to the square of height in meter square was used to determine the body mass index (BMI). Hypertension was defined as having an elevated average BP of two measures taken at least 14 days apart (SBP of 140 mmHg and/or DBP of 90 mmHg) or being on antihypertensive drugs.

Statistical analysis

Data analysis was done using STATA version 16.0 (StataCorp LLC, College Station, TX). Mean and standard deviations were reported for continuous variables, while frequency and percentage were reported for categorical variables. To determine the association between independent variables and hypertension, a univariate analysis was done using an independent t-test and chi-square test for continuous and categorical variables, respectively. At univariate analysis, p-value < 0.25 was considered significant. Variables significant at univariate analysis were used to make the final model through multivariable logistic regression. Finally, variables in the multivariable analysis with a p-value less than 0.05 were considered statistically significant, and an adjusted odds ratio (AOR) with a 95% confidence interval was calculated to assess the strength of the associations.

The article "Determinants of Hypertension Among Patients With Type 2 Diabetes Mellitus in Karachi, Pakistan: A Cross-Sectional Study" was retracted in 2022. Reasons: false authorship; lack of ethics approval or compliance; concerns about the data; concerns about the authorship.

## Results

A total of 610 patients were included in the study. Table 1 shows the demographic characteristics of participants. The mean age of participants was 57.37 (±11.32) years. The majority of study participants were females (50.33%), married (72.30%), and employed (65.08). More than one-quarter of participants (34.10%) had a family history of hypertension.

**Table 1:** Sociodemographic characteristics of participants. * Mean (standard deviation).

Variable	Categories	n (%)
Age*		57.37 (11.32)
Gender	Male	303 (49.67)
	Female	307 (50.33)
Marital status	Single	26 (4.26)
	Married	441 (72.30)
	Divorced	61 (10.00)
	Widowed	82 (13.44)
Employment	Unemployed	213 (34.92)
	Employed	397 (65.08)
Duration of diabetes	Less than 5 years	129 (21.15)
	5-10 years	174 (28.52)
	More than 10 years	307 (50.33)
Smoking status	Never	215 (35.25)
	Ex-smoker	224 (36.72)
	Current smoker	171 (28.03)
BMI	Underweight	5 (0.82)
	Normal	249 (40.82)
	Overweight	251 (41.15)
	Obese	105 (17.21)
Family history of hypertension	No	402 (65.90)
	Yes	208 (34.10)

Prevalence of hypertension among diabetes patients

The overall prevalence of hypertension among diabetic patients was found to be 39.84%. Table 2 shows the characteristics of participants with or without hypertension. The mean age was significantly higher in patients with hypertension (60.99 ± 10.02) than without hypertension (54.98 ± 11.36). Nearly half of the patients with hypertension had a family history of hypertension (47.33%), and it was significantly higher in patients without hypertension (25.43%). A sedentary lifestyle of more than four hours per day was reported in 45.27% of patients with hypertension and 31.06% in patients without hypertension. Among all the participants, the frequency of overweight and obesity was significantly higher in patients with hypertension than patients without hypertension.

**Table 2:** Comparison of sociodemographic characteristics between patients with hypertension and patients without hypertension. * Significant at p-value < 0.05. ^ Mean (standard deviation).

Variable	Categories	Hypertension		P-value
		Yes, n (%)	No, n (%)	
Age^		60.99 (10.02)	54.98 (11.36)	0.001*
Gender	Male	123 (50.62)	180 (49.05)	0.704
	Female	120 (49.38)	187 (50.95)	
Marital status	Single	12 (4.94)	14 (3.81)	0.007*
	Married	158 (65.02)	283 (77.11)	
	Divorced	28 (11.52)	33 (8.99)	
	Widowed	45 (18.52)	37 (10.08)	
Employment	Unemployed	90 (37.04)	123 (33.51)	0.372
	Employed	153 (62.96)	244 (66.49)	
Duration of diabetes	Less than 5 years	38 (15.64)	91 (24.80)	0.001*
	5-10 years	55 (22.63)	119 (32.43)	
	More than 10 years	150 (61.73)	157 (42.78)	
Smoking status	Never	52 (21.40)	163 (44.41)	0.001*
	Ex-smoker	103 (42.39)	121 (32.97)	
	Current smoker	88 (36.21)	83 (22.62)	
BMI	Underweight	2 (0.82)	3 (0.82)	0.003*
	Normal	80 (32.92)	169 (46.05)	
	Overweight	106 (43.62)	145 (39.51)	
	Obese	55 (22.63)	50 (13.62)	
Family history of hypertension	No	128 (52.67)	274 (74.66)	0.001*
	Yes	115 (47.33)	93 (25.43)	
Sedentary activity	≤4 hours	133 (54.73)	253 (68.94)	0.001*
	>4 hours	110 (45.27)	114 (31.06)	
Sleep duration	≤7.5 hours	112 (46.09)	163 (44.41)	0.684
	>7.5 hours	131 (53.91)	204 (55.59)	
Stress	No or low stress	44 (18.11)	126 (34.33)	0.001*
	Moderate or high stress	199 (81.89)	241 (65.67)	
Salt consumption after diabetes	No change in consumption	18 (7.41)	79 (21.53)	0.001*
	Minimally reduced	61 (25.10)	83 (22.62)	
	Substantially reduced	42 (17.28)	37 (10.08)	
	Stopped at all	122 (50.21)	168 (45.78)	
Physical activity	Low	113 (54.73)	160 (43.60)	0.008*
	Moderate	70 (28.81)	113 (30.79)	
	High	40 (16.46)	94 (25.61)	

Table 3 shows the laboratory values of participants. Median serum creatinine levels and median total cholesterol levels were significantly higher in patients with hypertension than patients without hypertension.

The article "Determinants of Hypertension Among Patients With Type 2 Diabetes Mellitus in Karachi, Pakistan: A Cross-Sectional Study" was retracted in 2022. Reasons: false authorship; lack of ethics approval or compliance; concerns about the data; concerns about the authorship.

**Table 3:** Comparison of laboratory parameters between patients with hypertension and patients without hypertension. * Significant at p-value < 0.05. Presented as median (interquartile range).

Variables	Hypertension		P-value
	Yes	No	
Hemoglobin A1c (%)	8.4 (7-10)	8.6 (7.2-9.8)	0.624
Serum creatinine (mg/dl)	1.0 (0.8-1.2)	0.82 (0.7-1.1)	0.007*
Total cholesterol (mg/dl)	175 (139-214)	165 (131-226)	0.028*
Low-density lipoprotein (mg/dl)	110 (82-139)	106 (83-130.5)	0.293
High-density lipoprotein (mg/dl)	41 (33-51)	41 (34-49)	0.426

Determinants of hypertension among people with diabetes mellitus

Based on the p-value of the univariate analysis presented in Tables 2, 3, a total of 12 variables were significant and considered for the multivariable model. These variables were age, marital status, duration of diabetes, smoking status, BMI, family history of hypertension, sedentary activity, stress level, salt consumption after diabetes, level of physical activity, serum creatinine, and total cholesterol levels.

The article "Determinants of Hypertension Among Patients With Type 2 Diabetes Mellitus in Karachi, Pakistan: A Cross-Sectional Study" was retracted in 2022. Reasons: false authorship; lack of ethics approval or compliance; concerns about the data; concerns about the authorship.

The results of the multivariable model are presented in Table 4. The results identified age, physical activity, family history of hypertension, smoking status, BMI, sedentary lifestyle, stress level, and serum creatinine as independent determinants of hypertension among people with type 2 diabetes mellitus.

**Table 4:** Variables significantly associated with hypertension among type 2 diabetes patients (multivariable logistic regression). AOR = adjusted odds ratio.

Variable	Categories	AOR (95% CI)	P-value
Age		1.06 (1.03-1.08)	0.001
Physical activity	Low		
	Moderate	0.75 (0.51-1.11)	0.158
	High	0.58 (0.37-0.91)	0.017
Family history of hypertension	No		
	Yes	3.06 (2.06-4.57)	0.001
Smoking status	Never		
	Ex-smoker	2.33 (1.47-3.71)	0.001
	Current smoker	3.11 (1.91-5.09)	0.001
BMI	Normal		
	Underweight	0.82 (0.12-5.32)	0.711
	Overweight	1.54 (1.07-2.22)	0.021
	Obese	2.32 (1.46-3.70)	0.001
Sedentary activity	≤4 hours		
	>4 hours	1.58 (1.06-2.37)	0.024
Stress	No or low stress		
	Moderate or high stress	2.52 (1.60-3.96)	0.001
Creatinine		2.82 (1.41-5.64)	0.003

## Discussion

The overall prevalence of hypertension among type 2 diabetes patients was found to be 39.84%. This was inconsistent with past studies conducted in Taiwan (39%) [15], Bahrain (38%) [16], and Pakistan (40.45%) [17]. On the other hand, the current findings showed a higher prevalence of hypertension among patients with type 2 diabetes than studies conducted in India (25.6%) [18] and Turkey (29%) [19]. Differences in socio-demographic, study design, kind of study population, sample size variation, and/or awareness differences could be explanations for discrepancies with our findings.

The current study shows that obesity is associated with hypertension among type 2 diabetes patients, which is consistent with the findings of a previous study [12]. The association is possibly because adipocytes in individuals with obesity cause the angiotensinogen activation that again raises sodium reabsorption and overload of volume in the renal system [20]. The increase in free fatty acids, which can cause hypertension either by its effect on the renal system or by generating inflammation, is another way obesity causes hypertension in obese people. Endothelial dysfunction is caused by inflammation, which results in vasoconstriction and arterial stiffness, which can lead to hypertension [21]. Besides this, when a person becomes overweight or obese, they will have excess bad cholesterol and insulin resistance, and it also makes blood vessels narrow, and gradually a person develops hypertension [21].

A sedentary lifestyle was also found to be an independent determinant of hypertension among type 2 diabetes patients. The findings of this study are supported by a cross-sectional study conducted at a hospital in Hosaena, Ethiopia [22]. The fact that persons who stay in a sedentary state have less physical activity exposes them to unhealthy weight gain, which leads to hypertension, could be a possible rationale for the link between sedentary behavior and hypertension [23].

The article "Determinants of Hypertension Among Patients With Type 2 Diabetes Mellitus in Karachi, Pakistan: A Cross-Sectional Study" was retracted in 2022. Reasons: false authorship; lack of ethics approval or compliance; concerns about the data; concerns about the authorship.

The current study showed that increasing age is an independent predictor of hypertension among type 2 diabetes patients. The findings of this study are inconsistent with the past studies [24,25]. This could be because aging is linked to deterioration in different physiological systems as well as non-communicable disorders like hypertension. Furthermore, growing older has been related to an increased risk of disease [12].

Besides this, the current study also showed that family history of hypertension is also an independent predictor of hypertension among type 2 diabetes patients. It means that odds of hypertension were higher in individuals having a family history of hypertension as compared to their counterparts. The findings of this study are supported by the study conducted by Kotiso et al. [26]. It is believed that several genetic factors are responsible for the development of hypertension along with environmental factors [27]. Therefore, individuals with a family history of hypertension are at higher risk of developing hypertension.

One of the main strengths of this study is unlike past studies conducted in Pakistan, this study included several confounders such as laboratory measurements, stress levels, and sedentary lifestyles. However, the current study has certain limitations like recall bias. It might be possible that the odds ratio for certain independent variables might be underestimated in the current study as patients started to exercise more after developing hypertension that underestimated the odds ratio of exercise. Because the study was conducted in a hospital, it may not be representative of the general public, and certain questions were subjected to recall bias. Finally, concurrent drugs were not taken into account.

## Conclusions

In this study, age, physical activity, family history of hypertension, smoking status, BMI, sedentary lifestyle, stress level, and serum creatinine are independent determinants of hypertension among type 2 diabetes patients. The findings of the study call for strategies that can target these predictors, and clinicians need to start educating their patients about hypertension and ways to prevent it. Besides this, policymakers need to develop policies at the individual and collective levels to increase the physical activity level of employees.
